# Risk factors for post-ERCP pancreatitis: a systematic review of clinical trials with a large sample size in the past 10 years

**DOI:** 10.1186/2047-783X-19-26

**Published:** 2014-05-15

**Authors:** Jian-Jun Chen, Xi-Mo Wang, Xing-Qiang Liu, Wen Li, Mo Dong, Zong-Wu Suo, Po Ding, Yue Li

**Affiliations:** 1 Department of Gastroenterology, Tianjin Nankai Hospital, No.6 Changjiang Road Nankai District, Tianjin 300100, China; 2 Department of Gastroenterology, People's Hospital of Tianjin, Jieyuan Road 190, Tianjin 300121, China

**Keywords:** Endoscopic retrograde cholangiopancreatography, Pancreatitis, Risk factors, Systematic review

## Abstract

**Background:**

Post- endoscopic retrograde cholangiopancreatography (ERCP) pancreatitis (PEP) is the most common and most severe complication associated with diagnostic and therapeutic ERCP. A multivariate analysis of risk factors for PEP is essential for identifying patients at high risk and subsequently choosing other suitable diagnoses.

**Methods:**

Pertinent publications were identified through systematic searches of MEDLINE, Elsevier, and Springer; we performed a systematic review of 12 clinical studies published in the past ten years, selected out of 451 reviewed articles, in which risk factors for pancreatitis were identified. Seven probable risk factors were evaluated, and outcomes expressed in the case of dichotomous variables, as an odds ratio (OR) (with a 95% confidence interval, 95% CI).

**Results:**

When the risk factors were analyzed, the OR for female gender was 1.40 (95% CI 1.24 to 1.58); the OR for previous PEP was 3.23 (95% CI 2.48 to 4.22); the OR for previous pancreatitis was 2.00 (95% CI 1.72 to 2.33); the OR for endoscopic sphincterotomy was 1.42 (95% CI 1.14 to 1.78); the OR for precut sphincterotomy was 2.11 (95% CI 1.72 to 2.59); the OR for Sphincter of Oddi dysfunction was 4.37 (95% CI 3.75 to 5.09); and the OR for non-prophylactic pancreatic duct stent was 2.10 (95% CI 1.63 to 2.69).

**Conclusions:**

It appears that female gender, previous PEP, previous pancreatitis, endoscopic sphincterotomy, precut sphincterotomy, Sphincter of Oddi dysfunction, and non-prophylactic pancreatic duct stent are the risk factors for post-ERCP pancreatitis.

## Background

Since endoscopic retrograde cholangiopancreatography (ERCP) was first introduced in 1968, it has been performed as a diagnostic and therapeutic procedure for various biliary and pancreatic diseases. The role of ERCP changed from a diagnostic modality to a therapeutic procedure after the introduction of recent developments in magnetic resonance cholangiopancreatography (MRCP) [1]. Post-ERCP pancreatitis (PEP) is the most common and severe complication associated with diagnostic and therapeutic ERCP [2-4]. A small percentage of patients may develop severe pancreatitis resulting in a prolonged hospitalization, intensive care unit admission and utilization of major hospital resources; these patients have a significant morbidity and mortality [5]. The incidence of PEP reached up to 3.5% in a systematic review of 21 clinical studies [6]. While the technology and equipment of ERCP continue to improve, how to reduc the occurrence of PEP is still a serious clinical problem. It is useful to identify exactly which conditions are related to this complication, in order to avoid PEP in patients in whom protective endoscopic or pharmacological measures should be considered. There is still controversy concerning the risk factors related to PEP. The aim of the present study was to perform a systematic review of a series of cases of PEP to compare the risk factors predisposing to this complication which have been mentioned in the literature.

## Methods

### Identification of trials

Inclusion criteria were as follows [7]: 1) primary clinical data about multivariate analysis of risk factors for post-ERCP pancreatitis in the past ten years; 2) criterion in determining the diagnosis of post-ERCP pancreatitis: there was at least a three-fold increase in serum amylase concentration occurring 24 hours after an ERCP, accompanied with obvious abdominal pain; and 3) the literature data were reliable, and the full text could be obtained.

Exclusion criteria were as follows: 1) retrospective analysis contained less than 100 cases (the proficiency of surgeons has a great impact on the results in clinical research with a small sample size); 2) the article types were either review or case report; 3) there were only OR values and 95% CI instead of original data in the articles; 4) duplication of results; and 5) studies with less information or unknown data description.

### Data search strategy

To obtain relevant clinical studies in English and Chinese, a systematic literature search with predefined search terms was carried out in MEDLINE, Elsevier and Springer links. or articles published between 2002 and 2012. The predefined search terms were ‘ERCP (endoscopic retrograde cholangiopancreatography)’, ‘pancreatitis’, and ‘risk factors’. The reference lists of all pertinent reviews and articles were checked to identify additional studies not found in the computerized database search.

### Data extraction and quality assessment

Two authors independently read the abstracts of retrieved articles and, subsequently, full-text articles to identify whether the data were suitable for the systematic review on the basis of specified inclusion and exclusion criteria. Discrepancies in selection were resolved by discussion.

The Jadad scale [8] was used to grade the methodological quality of the trials included. The quality scale ranges from 0 to 5 points, with two or less indicating low quality and three or more indicating high quality.

### Statistical analysis

To obtain a global measure of the comparative data, meta-analytical techniques based on The Cochrane Collaboration’s Review Manager (RevMan version 4.2) were used. The estimation of count data is expressed, in the case of dichotomous variables, as an odds ratio (OR) (with a 95% confidence interval, 95% CI). *P* <0.05 was deemed statistically significant difference.

## Results

### Description of studies

We reviewed 451 articles that met our search criteria. After rigorous screening of their full text, 12 of them satisfied the study inclusion criteria and were included (Table 1) [3,9-19].

**Table 1:** Description of the 13 included studies

**Study**	**Year**	**Number**	**Methods**	**Incidence of PEP**	**The rates of therapeutic procedures**
Andriulli (9)	2002	579	RCT, multicenter, paralled group	8.64%	Nr
Vandervoort (17)	2002	1,223	Single center, prospective analysis	7.20%	54.7%
Perney (13)	2003	173	Single center, retrospective analysis	17.92%	Nr
Andriulli (10)	2004	1,127	RCT, multicenter, paralled group	5.59%	Nr
Xia (12)	2004	380	Single center, retrospective analysis	4.47%	73.7%
Cheng (11)	2006	1,088	RCT, multicenter, paralled group	15.44%	51.9%
Tsuyuguchi (16)	2007	184	Single center, prospective analysis	1.09%	79.9%
Cotton (3)	2009	11,497	Single center, retrospective analysis	2.64%	Nr
Matsubayashi (14)	2009	740	Single center, retrospective analysis	3.92%	Nr
Wilox (18)	2010	3,499	Single center, prospective analysis	3.15%	Nr
Testoni (15)	2010	3,635	Multicenter, prospective analysis	3.77%	96.6%
Zhou (19)	2011	7,168	Single center, retrospective analysis	3.70%	NR

### Results of risk factor evaluation

In total, there were 32,381 post-ERCP patients involved in this review, and 1,309 of them suffered PEP. The incidence of PEP was 4.04%. The following were considered as risk factors and related information was extracted and analyzed: sex, history of previous PEP, history of previous pancreatitis, endoscopic sphincterotomy (EST), precut sphincterotomy, Sphincter of Oddi Dysfunction (SOD) and pancreatic duct stenting.

### Participants

Eleven studies reported the influence of gender on PEP. The incidence of PEP in female patients was 4.47%, compared with 3.22% in male patients. The risk of the occurrence of PEP in women was 50% more than that of men, and the difference was statistically significant (*P* <0.01). The results of the systematic review are shown in Figure 1.

**Figure 1:** The effect of female/male gender.

### Previous PEP

Six studies reported patients with previous PEP. The incidence of PEP in these patients was 17.82%, compared with 5.03% in control patients. There was a 2.23 times increased incidence for patients with previous PEP, and the difference was statistically significant (*P* < .01). The results of the systematic review are shown in Figure 2.

**Figure 2:** The effect of previous PEP.

### Previous pancreatitis

Eight studies reported patients who had a history of previous pancreatitis. The incidence of PEP in these patients was 5.46%, compared with 3.12% in control patients. The risk of the occurrence of PEP is increased one-fold, and the difference was statistically significant (*P* <0.01). The results of the systematic review are shown in Figure 3.

**Figure 3:** The effect of previous pancreatitis.

### Endoscopic sphincterotomy (EST)

Eight studies reported patients who underwent an endoscopic sphincterotomy. The incidence of PEP in these patients was 7.09%, compared with 5.50% in control patients. The risk of the occurrence of PEP in patients with EST increased by 42%, and the difference was statistically significant (*P* <0.01). The results of the systematic review are shown in Figure 4.

**Figure 4:** The effect of endoscopic sphincterotomy.

### Precut sphincterotomy

Nine studies reported patients operated on using the precut technique. The incidence of PEP in these patients was 9.64%, compared with 4.93% in control patients. There was a 1.11 times increased incidence with the precut technique, and the difference was statistically significant (*P* <0.01). The results of the systematic review are shown in Figure 5.

**Figure 5:** The effect of precut sphincterotomy.

### Sphincter of Oddi dysfunction

Nine studies reported patients with SOD. The incidence of PEP in these patients was 9.74%, compared with 3.11% in control patients. There was a 3.37 times increased incidence for SOD, and the difference was statistically significant (*P* <0.01). The results of the systematic review are shown in Figure 6.

**Figure 6:** The effect of Sphincter of Oddi dysfunction.

### Non-prophylactic pancreatic duct stent

Three studies reported patients who underwent pancreatic duct stenting. The incidence of PEP in these patients was 10.21%, compared with 4.12% in control patients. There was a 1.1 times increased incidence for pancreatic duct stenting, and the difference was statistically significant (*P* <0.01). The results of the systematic review are shown in Figure 7.

**Figure 7:** The effect of pancreatic duct stenting.

## Discussion

ERCP is the procedure of choice for treating biliary tract and pancreatic diseases. While the technology and equipment of ERCP continue to improve, postoperative complications cannot be completely avoided due to the invasive form of this surgery. PEP was the most serious and common complication following ERCP. How to determine risk factors for PEP is an all too urgent clinical issue because it is essential for identifying patients at high risk and subsequently choosing other suitable treatment, such as magnetic resonance cholangiography, endoscopic ultrasonography, percutaneous transhepatic biliary drainage, and so on.

After rigorous screening, 13 clinical trials which provided data about risk factors for PEP were included in this systematic review. The results suggest that female gender, previous PEP, previous pancreatitis, precut sphincterotomy, SOD and so on were all risk factors for PEP.

It is difficult to demonstrate whether female gender is an independent risk factor. The increased incidence of PEP in women would probably be because SOD affects women more frequently than men [12].

EST s a common and essential procedure in therapeutic ERCP. Akashi *et al*. [20] reported that the edema in surrounding tissues was induced because of the sensitivity of the pancreatic duct to thermal damage caused by EST and subsequently the pancreatic duct was temporarily blocked, all of which caused the occurrence of PEP. However, in many studies [21-24], EST was not considered to be a risk factor for PEP. Theoretically, EST can reduce the tension at the orifice of the pancreatic duct. The incidence of post-EST pancreatitis is largely dependent upon the skill of the endoscopist, in addition to factors related to the host. Endoscopists must aim to improve their technique and fully utilize their abilities under an adequate guidance system [25].

Precut sphincterotomy may cause edema of the duodenal papilla, a poor discharge of pancreatic juice,and induce post-ERCP acute pancreatitis [26]. In this study, the incidence of PEP in patients after precut sphincterotomy was approximately twice that in patients without precut sphincterotomy. Some studies showed that the incidence of complications after precut sphincterotomy was closed is related to the precut position, and that there is a minimal risk for postoperative complications when the precut occurs on the top of the duodenal papilla [19]. Thus, the top of the papilla is a better choice for precut sphincterotomy. Pre-cut techniques are mostly used after conventional methods of biliary cannulation have failed or, in a few centers, as a preferential technique for performing biliary and pancreatic sphincterotomy over a pancreatic stent in patients with SOD [27]. Therefore, difficult cannulation is a risk factor for PEP. Martin *et al*. [28] reported that the incidence of PEP after precut sphincterotomy is highly related to the technique used by the endoscopists. Further research is necessary to access the relationship between pre-cut techniques and PEP.

SOD is a benign noncalculous obstructive disorder occurring at the level of the Sphincter of Oddi which causes pancreaticobiliary-type pain. Criteria for diagnosing SOD have been established by the Rome III conference [29]. Patients suspected of having SOD should have episodes of abdominal pain that is located in the epigastrium and right upper quadrant and is associated with the following features: 1) ≥30 minutes in duration, 2) recurrent symptoms occurring at variable intervals (not daily), 3) occurring on one or more occasions in the last 12 months, 4) pain that builds up to a steady level, 5) pain that is moderate to severe enough to interrupt a patient's daily activities, and 6) no evidence of structural abnormalities to explain the symptoms. SODis more common in women. SOD is considered a definite independent risk factor for PEP in some studies [18-20]. The placement of a pancreatic stent or nasal pancreatic drainage would significantly reduce the incidence of PEP in patients with SOD.

Recently, research supported pancreatic-stent placement as an effective intervention for the prevention of PEP in high-risk patients [30]. However, placement of a pancreatic-stent is a risk factor for PEP in this systematic review. This is mainly because the pancreatic-stent placement was for therapeutic purposes other than prevention in the included studies. Patients with pancreatic diseases, such as obstruction of the pancreatic duct and pancreatolithiasis, needed drainage of pancreatic juice via a pancreatic stent.

A similar study was reported by Masci *et al*. in 2003 [7], which showed that the risk factors for PEP may change according to the development of instruments and technologies. Therefore we chose more potential risk factors in this systematic review of clinical trials in the past ten years, which would give a more objective response of risk factors for PEP.

From this systematic review a three-pronged approach could be advised to prevent PEP: 1) Preoperative examination is needed to determine patients who are suitable to undergo surgery; 2) Surgeons need more suitable training to improve their surgical proficiency; and 3) Various preoperative, intraoperative and postoperative preventive practices should be used, such as the use of somatostatin analogs [31] and pancreatic stents [30], could minimize the incidence of PEP and reduce harm to patients.

The limited information in some studies, the absence of some variables, the fact that many risk factors had already been identified in previous studies, and the fact that many were reported in a way that precluded comparison across studies may limit the usefulness of our results. However, the large number of cases considered for analysis of the single risk factors for pancreatitis substantiate the findings.

Several limitations of the present study need to be considered. First, it is difficult to perform randomized controlled trials (RCTs) because of the low incidence of PEP, so both prospective and retrospective studies were selected for analysis, which produces some bias in the analysis. Secondly, there was significant heterogeneity among these studies. The heterogeneity might be explained by the study design, study quality, patients’ characteristics, and the diverse technical specifications.

## Conclusions

Despite these limitations, our findings have important implications concerning the risk factors for PEP, and we conclude that female gender, previous PEP, previous pancreatitis, endoscopic sphincterotomy, precut sphincterotomy, SOD and non-prophylactic pancreatic duct stent are the risk factors for post-ERCP pancreatitis.

## Abbreviations

CI: confidence interval; ERCP: endoscopic retrograde cholangiopancreatography; OR: odds ratio; PEP: post-ERCP pancreatitis; EST: endoscopic sphincterotomy; SOD: Sphincter of Oddi dysfunction.

## Competing interests

The authors declare the have no competing interest.

## Authors' contributions

JJC and XMW defined the research theme; XQL, WL and MD co-worked on associated data collection; ZWS, PD and YL discussed analyses; JJC and XMW wrote the paper. All authors read and approved the final manuscript.
